RETRACTED

# Myocardial ischemia reperfusion injury is alleviated by curcumin-peptide hydrogel via upregulating autophagy and protecting mitochondrial function

**DOI:** 10.1186/s13287-020-02101-y

**Published:** 2021-01-28

**Authors:** Chi-Lin Liao, Yang Liu, Meng-Zhao Huang, Hua-Yong Liu, Zi-Liang Ye, Qiang Su

**Affiliations:** 1 Department of Cardiology, People’s Hospital of Baise, Baise, 533000 People’s Republic of China; 2 Department of Cardiology, The Second People’s Hospital of Nanning City, The Third Affiliated Hospital of Guangxi Medical University, Nanning, 530031 People’s Republic of China; 3 Department of Cardiology, Affiliated Hospital of Guilin Medical University, No. 15, Lequn Road, Xiufeng District, Guilin, 541001 Guangxi Zhuang Autonomous Region People’s Republic of China

**Keywords:** Ischemia-reperfusion injury, Autophagy, Apoptosis, Curcumin, Hydrogel

## Abstract

**Background:**

Ischemia-reperfusion injury (IRI) is an important factor limiting the success of cardiac reperfusion therapy. Curcumin has a significant cardioprotective effect against IRI, can inhibit ventricular remodeling induced by pressure load or MI, and improve cardiac function. However, the poor water solubility and low bioavailability of curcumin restrict its clinical application.

**Methods:**

In this study, we prepared and evaluated a curcumin-hydrogel (cur-hydrogel) to reduce cardiomyocyte apoptosis and reactive oxygen species formation induced by hypoxia-reoxygenation injury, promote autophagy, and reduce mitochondrial damage by maintaining the phosphorylation of Cx43.

**Results:**

Meanwhile, cur-hydrogel can restore cardiac function, inhibit myocardial collagen deposition and apoptosis, and activate JAK2/STAT3 pathway to alleviate myocardial ischemia-reperfusion injury in rats.

**Conclusions:**

The purpose of this study is to elucidate the protective effects of cur-hydrogel on myocardial ischemia-reperfusion injury by regulating apoptosis, autophagy, and mitochondrial injury in vitro and in vivo, which lays a new theoretical and experimental foundation for the prevention and reduction of IRI.

## Background

The reperfusion therapy of acute myocardial infarction can lead to more serious dysfunction after myocardial ischemia, resulting in the decrease of myocardial diastolic and systolic function, the decrease of ventricular threshold, and the shortening of refractory period, which can be manifested as malignant arrhythmia, cardiac insufficiency, and even sudden death [1, 2]. The mechanism of ischemia-reperfusion injury is not completely clear. At present, the mechanisms with more evidence include oxidative stress, intracellular calcium overload, vascular endothelial injury, endoplasmic reticulum stress, and inflammatory response [3, 4]. To develop effective drugs or treatments to reduce myocardial ischemia-reperfusion injury has become a key problem to be solved urgently.

RETRACTED

Curcumin is a polyphenolic compound extracted from the rhizome of curcuma. As an effective ingredient of traditional Chinese medicine turmeric, curcumin has a variety of pharmacological effects, such as anti-inflammation, anti-oxidation, anti-apoptosis, anti-fibrosis, anti-tumor, cardiovascular protection, and so on. Studies have shown that curcumin has a protective effect on myocardial ischemia-reperfusion injury and can reduce oxidative stress injury and cardiomyocyte apoptosis [5]. Curcumin can also inhibit angiotensin II-mediated myocardial fibrosis [6] and cardiac non-benign ventricular remodeling caused by left ventricular pressure overload [7] by regulating the expression of angiotensin receptor. It can also reduce myocardial hypertrophy caused by diabetic cardiomyopathy and improve cardiac function [8]. Curcumin can also improve the cardiac function of rats after myocardial infarction in a dose-dependent manner [9] and can prevent the progression of heart failure after myocardial infarction [10]. In the treatment of heart failure, curcumin can inhibit myocardial fibrosis and inhibit the activation of myocardial fibroblasts by regulating TGF-β/Smads signaling pathway to reduce collagen synthesis and reduce ventricular remodeling after heart failure [11]. However, curcumin has poor water solubility, easy oxidation in vitro, and low bioavailability. For example, in the human pharmacokinetic test, volunteers take a large dose of curcumin 12 g per day, but the blood concentration is too low to be detected, and its metabolic degradation is very fast. These shortcomings seriously restrict the wide clinical application of curcumin [12, 13].

In order to increase the water solubility and bioavailability of curcumin, various dosage forms of curcumin carriers have been developed, such as polymer nanoparticles, polymer micelles, microemulsions, microspheres, liposomes, and polymer hydrogels [14]. These carriers greatly improve the water solubility and bioavailability of curcumin by encapsulation, chemical bond linking, or physical adsorption. The degradation products of small molecular hydrogels of polypeptides are amino acids, which have the advantages of easy degradation, high biocompatibility, non-toxicity, and safety, and have been widely used in biological fields such as three-dimensional cell culture, drug controlled release, biosensor, and so on. At present, cur-hydrogels are mainly made of high molecular hydrogels (such as galactose, chitosan, gelatin, chitin, and polyacrylamide gelatin) or covalently linked to cur-hydrogels [15]. It has been studied that polypeptide Nap-GFFYG-RGD and curcumin monomer were assembled into small molecular polypeptide hydrogel, which significantly improved the anti-tumor effect [16].

RETRACTED

In this study, we prepared a kind of hydrogel as curcumin carrier in order to improve the bioavailability of curcumin. We hypothesize that cur-hydrogel may have a better therapeutic effect on heart ischemia-reperfusion injury and explore its mechanism.

## Methods

### Animals

Healthy male SD rats were selected and fasted 12 h before the animal experiment. The rats were anesthetized by pentobarbital sodium according to their body weight. The ECG were monitored and recorded by electrocardiograph.

Cut the skin of the rat neck with aseptic scissors, fully expose the trachea, intubate the trachea with an indwelling needle, connect the small animal ventilator, give artificial ventilation (pressure 3kpa, frequency 70 times/min) to assist breathing, open the chest in the left fifth auxiliary room beside the sternum, separate the pericardium, fully expose the heart, the left coronary artery is located between the left atrial appendage and the pulmonary artery, and use a small curved needle at 1–2 mm under the left atrial appendage. The left anterior descending branch of the coronary artery was ligatured at the upper 1/3 of the left anterior descending branch (note that the needle depth was not more than 1 mm, and the width was not more than 3 mm). The color of the anterior wall of the distal end of the coronary artery was observed to become purplish red. ECG monitoring showed that the ST segment in lead I, II, avL of ECG elevated 0.2 mV as a sign of successful operation. 40 μM, 20 μL curcumin or cur-hydrogel was injected to ventricular wall at the bilateral 1 mm of the ligation site with an insulin injection needle (30 G), and then, the chest was closed and sutured. AG490 (3 mg/kg) was injected intraperitoneally 30 min before operation in the model of heart injury. This study has been approved by the Animal Experimental Ethics Committee of Affiliated Hospital of Guilin Medical University and was carried out in accordance with the National Institutes of Health guide for the care and use of Laboratory animals (NIH Publications No. 8023, revised 1978). The rats were raised in the SPF animal room of the Clinical Research Center of the Affiliated Hospital of Guilin Medical University, feeding standard chow diet with light-dark cycle for 12 h. After the termination of experiments, the rats were euthanized by an anesthetic overdose.

### Cardiac hemodynamic measurement

A small latex balloon filled with water was inserted into the left atrium by polyethylene intubation and entered into the left ventricle. The pressure transducer was connected to measure the left ventricular diastolic pressure (LVDP), left ventricular end-diastolic pressure (LVEDP), and the maximum rate of rise and fall of left ventricular pressure. The data were input into the computer to analyze and record them.

RETRACTED

### Cardiac ultrasound examination of cardiac function

Five mice in each group were randomly selected for cardiac ultrasound 4 weeks after surgery. After intraperitoneal injection of pentobarbital sodium, the mice were fixed on a constant temperature plate at 37 °C. The chest was evenly smeared with ultrasonic coupling agent and detected by Mindray DP-50 ultrasound system. Each mouse was measured for 10 consecutive cardiac cycles and the left ventricular ejection fraction (LVEF) and left ventricular short axis shortening rate (LVFS), LVEF = [(LVEDV-LVESV)/LVEDV] × 100%, LVFS = [(LVEDD-LVESD)/LVEDD] × 100%.

### Evans blue staining

The coronary artery was ligated in situ, and retrograde perfusion was performed through the aorta with 2–3 ml Evans Blue (1%) under a certain pressure (80 mmHg). Under the action of staining, the non-ischemic heart showed blue, which supported the display of ischemic AAR (risk zone) myocardium.

### HE/Masson staining

The experimental animals were euthanized by injecting excessive pentobarbital sodium. The heart was removed immediately, and part of the myocardial tissue was fixed in paraformaldehyde, and ethanol was used for gradient dehydration, followed by transparent treatment and paraffin embedding. After the embedded myocardial tissue was cooled and solidified, it was cut into thin slices with a thickness of 5 μm. The myocardial tissue of rats was stained with HE (hematoxylin-eosin staining) and collagen was stained with Masson.

### Determination of biochemical indexes of myocardial tissue

The myocardial tissue was homogenized at 60 Hz for 60 s for 2 times in an automatic sample grinder, and the supernatant was centrifuged at 3500 r/min for 10 min at 4 °C. The samples were separated and stored in the refrigerator at − 80 °C for the determination of content and the activities of SOD, CAT, and GPS,GR, respectively. After strictly following the instructions of the kit, the OD values were determined by enzyme labeling instrument.

### Enzyme colorimetric method

The activities of Ca^2+^-ATPase and Na^+^-K^+^-ATPase in aorta were determined by enzyme colorimetry (Nanjing Jiancheng Institute of Biological Engineering, China). Strictly according to the instructions of ultra-trace Ca^2+^-ATPase and Na^+^-K^+^-ATPase detection kit, the activities of enzyme in myocardial tissue homogenate were determined.

RETRACTED

### Preparation of cur-hydrogel

The peptide RADA16-I (Ac-RADARADARADARADA-CONH2) stored at 4 °C and was synthesized by Shanghai Bootech BioScience & Technology (Shanghai, China).

The method of configuration of curcumin-RADA16-I solution was as follows: appropriate curcumin and RADA16-I were placed in 10 ml vials, and water was added to vials, obtaining curcumin solution with concentration of 5.0 × 10^3^ M and RADA16-I solution with concentration of 5.8 × 10^5^ M (0.1 mg/ml). The solution is left in a mixing pan for about 5 days.

### Dynamic light scattering (DLS)

The particle size distribution of the cur-hydrogel suspension was measured by dynamic light scattering particle size analyzer (Nano-ZS90, Malvern, UK). The suspension is shaken vigorously before measurement.

### Drug release kinetics in vitro

Under the simulated environment of physiological temperature in vitro, the release time and rate of curcumin from co-assembled hydrogel were observed. It was detected by high-performance liquid chromatography-mass spectrometry (LC-MS).

### Hypoxia-reoxygenation model of cardiomyocytes

H9C2 cardiomyocytes (Boster Biological Technology, Wuhan, China) were cultured in DMEM medium containing 10% serum (GIBCO, USA) and 1% penicillin-streptomycin at 37 °C and 5% CO_2_ incubator. According to the experimental group, the original complete culture medium was replaced by serum-free low-sugar DMEM medium, and H9C2 cardiomyocytes were placed in an anoxic incubator with 37 °C, 5% CO_2_, and 2% O_2_ for 12 h. After hypoxia, the culture medium was replaced by complete culture medium and reoxygenated in an incubator of 37 °C and 5% CO_2_ for 12 h to establish a cell HR model.

### MTT assay

H9C2 cells were plated in 96-well plates and we used MTT assay to detect the cell viability. MTT (0.5 mg/mL, Beyotime Biotechnology, China) was added after curcumin treatment and incubated for 3 h at 37 °C. And 150 μL DMSO was added and incubated for 15 min. We measured the absorbance at 490 nm.

### Flow cytometry

The Annexin V-FITC/PI apoptosis detection kit was purchased from Solebao Company (Beijing, China), and an appropriate amount of logarithmic growth phase cells were washed twice with pre-cooled PBS. The cells were suspended with 500 ul of bound buffer, mixed with 5 μl of annexin V-FITC and PI, respectively, and placed at room temperature for 15 min. The apoptosis rate was determined by flow cytometry.

### Single fluorescent GFP-LC3 plasmid transfection

After transient transfection of GFP-LC3 plasmid into H9C2 cells, the changes of green bright spots of GFP-LC3 in each group were observed under double fluorescence microscope, and 5 visual fields were randomly selected in each experimental group to take pictures.

RETRACTED

### TUNEL staining

According to the instructions, the cells or tissues were successively added with biotin labeling solution and 3,3-diaminobenzidine carbon tetrachloride (DAB) chromogenic solution and used PBS. Finally, the 3DHISTECH Pannoramic SCAN system was used to scan 5 non-overlapping visual fields in each group. The apoptotic nuclei and the total number of apoptotic nuclei in the visual field were calculated by Image J software. The apoptosis rate of cardiomyocytes = the number of apoptotic nuclei/the total number of nuclei × 100%.

### DCFH-DA probe staining

DCFH-DA probe (Sigma, USA) is used to detect the formation of reactive oxygen species. The cardiomyocyte culture medium was removed; diluted DCFH-DA (10uM) probe 1 ml was added and incubated at 37 °C in 5%CO_2_ incubator for 20 min. Rinse with PBS for 3 times × 1 min to fully remove the DCFH-DA probe that did not enter the cell. Then, the fluorescence intensity was detected by laser confocal microscope.

### Determination of mitochondrial membrane potential

JC-1 reagent (T3168) was purchased from Semel Fisher Technology Co., Ltd. (China). Strictly follow the instructions. 1 μg/mL JC-1 working solution was prepared and incubated at 37 °C for 20 min, PBS. Five visual fields were selected for each group and photographed under confocal microscope.

### Western blot

Take appropriate amount of cells in logarithmic growth phase, after RIPA cleavage, extract total protein, BCA method. After quantitative denaturation, protein electrophoresis-membrane transfer-closure-I anti-incubation-II anti-incubation-development exposure were carried out according to the operation steps. The expression of the target protein was expressed by the ratio of the gray value.

### Statistical analysis

All data is presented as a mean ± S.E.M. Statistical analysis was performed using a one-way ANOVA. *P* value < 0.05 was considered as statistically significant.

## Results

### Construction and characterization of cur-hydrogel

cur-hydrogel can form nanofibers with different thickness, the diameter is about 1000 nm (Fig. 1a), and interweave and winding each other to form a three-dimensional network structure. The cur-hydrogel has good mechanical properties and stability and can slowly release curcumin monomer in vitro (Fig. 1b).

**Fig. 1:** Characteristics of cur-hydrogel. **a**. DLS was used to detect the particle size of curcumin hydrosol. **b** The cumulative release amount of curcumin from hydrogel to PBS solution (37 °C pH 7.4)

### The protective effect of cur-hydrogel on cardiomyocyte injury induced by HR was better than curcumin

We treated the cells with different concentrations of curcumin or curcumin-loaded hydrogels (20, 40, 60 μM) for 24 h, followed by hypoxia-reoxygenation injury. MTT results showed that both curcumin group and curcumin-loaded hydrogel group had inhibitory effect on cell death, and the effect of cur-hydrogel group was better at the same concentration (Fig. 2a).

RETRACTED

**Fig. 2:** cur-hydrogel attenuated cardiomyocyte apoptosis induced by HR. **a** The effect of curcumin and cur-hydrogel on cell survival rate was evaluated by MTT. *n* = 5. **b** Apoptosis-related proteins were detected by western blot. *n* = 3, *p < 0.05; **p < 0.05. **c** Annexin V-FITC/PI apoptosis kit was used to detect cell apoptosis. *n* = 3, *p < 0.05; **p < 0.05. **d** TUNEL staining and statistical chart. (Bar = 150 μm) *n* = 5, *p < 0.05; **p < 0.05

We chose 40 μM curcumin group or curcumin-loaded hydrogel group to inhibit cell death. The results of flow cytometry (Fig. 2b) and TUNEL staining (Fig. 2c) showed that cur-hydrogel could reduce apoptosis better at the same concentration. The results of Western blotting showed that curcumin or curcumin-loaded hydrogel decreased the protein levels of Bid, Bax, caspase-3, and caspase-9 induced by hypoxia-reoxygenation, and the effect of cur-hydrogel was better than that of curcumin group (Fig. 2d).

As shown in Fig. 3a, both curcumin and cur-hydrogels can inhibit cell ROS production, and the effect of cur-hydrogel is better at the same concentration. The changes of p38 MAPK/NF-kB in ROS-related pathway were determined by Western blotting. Hypoxia-reoxygenation injury increased the expression of pamp T-p38 MAPK and NF-kB, while cur-hydrogel significantly decreased the expression of these proteins (Fig. 3b).

**Fig. 3:** cur-hydrogel inhibited the formation of reactive oxygen species induced by HR. **a** Detection of reactive oxygen species formation by DCFH-DA staining. (Bar = 75 μm) *n* = 3, *p < 0.05; **p < 0.05. **b** p-p38 MAPK and p-NF-kB protein levels were evaluated by western blot. *n* = 3, *p < 0.05

Curcumin has been reported to affect the level of autophagy. In this study, mRFP-GFP-LC3 adeno-associated virus was used to transfect H9C2 cardiomyocytes labeled LC3. As shown in Fig. 4a, the expression of autophagosomes decreased due to hypoxia-reoxygenation injury, and cur-hydrogel could promote autophagy more than curcumin. In Fig. 4b, the transformation of autophagy marker protein LC3-I to LC3-II was further detected by western blot, and the level of p62 protein was measured. Compared with curcumin, cur-hydrogel could promote the transformation from LC3-I to LC3-II and inhibit the expression of p62.

RETRACTED

**Fig. 4:** cur-hydrogel promoted autophagy of injured cardiomyocytes. **a** GFP-LC3 staining was used to assess autophagy (Bar = 25 μm). **b** p62 and LC3 protein levels were analyzed by western blot. *n* = 3, *p < 0.05

We used JC-1 probe to detect the degree of mitochondrial depolarization after cur-hydrogel treatment. In the HR group, the mitochondrial membrane potential decreased (red fluorescence decreased). After curcumin treatment, the decrease of mitochondrial membrane potential was alleviated, and after cur-Hydrogel treatment, the decrease of mitochondrial membrane potential was further alleviated. Hydrogel had no effect on mitochondrial membrane potential as in the control group (Fig. 5a). Western blotting showed that p-Cx43/Cx43 ratio was decreased by HR treatment, p-Cx43/Cx43 ratio was improved by curcumin treatment, and p-Cx43/Cx43 ratio was further improved by cur-hydrogel group (Fig. 5b).

**Fig. 5:** cur-hydrogel restored mitochondrial function. **a** JC-1 staining was used to analysis mitochondrial membrane (Bar = 20 μm). **b** Protein level of Cx43 and phosphorylated Cx43 were assessed by western blotting. *n* = 3, *p < 0.05

### cur-hydrogel was superior to curcumin in relieving myocardial ischemia-reperfusion injury in rats

We established a rat model of myocardial ischemia-reperfusion and treated with curcumin or hydrogel curcumin. First of all, we measured the left ventricular diastolic blood pressure (LVDP), left ventricular end-diastolic pressure (LVEDP), and the maximum rate of rise and fall of left ventricular pressure (dp/dt max). The results showed that cur-hydrogel could significantly restore the cardiac function of model mice, and its effect was better than that of curcumin. (Table 1). Superoxide dismutase (SOD), catalase (CAT), glutathione peroxidase (GPX), and glutathione reductase (GR) coordinate to prevent excessive level of reactive oxygen species in cells, which is collectively referred to as protective enzyme system. cur-hydrogel can increase the activity of these enzymes more than curcumin and play a protective role in cardiomyocytes (Table 2). The activities of Ca^2+^-ATPase and Na^+^-K^+^-ATPase in myocardial sarcoplasmic reticulum were determined. cur-hydrogel could significantly restore the activity of Ca^2+^-ATPase and Na^+^-K^+^-ATPase in model mice (Table 3). The hydrogel treatment had no significant effect on the cardiac function of rats. However, with JAK2/STAT3 inhibitor AG490, the effect of cur-hydrogel was reversed. (Tables 1, 2, and 3).

**Table 1:** Changes of cardiac hemodynamics

Group	LVDP (mmHg)	LVEDP (mmHg)	+dp/dtmax (mmHg/s)	+dp/dtmin (mmHg/s)
**Sham**	**98.26 ± 8.59**	**1725 ± 15.36**	**1802.45 ± 157.24**	**1326.57 ± 100.78**
**IR**	61. 52 ± 25.92 *	1043.26 ± 98.25 *	1236.26 ± 118.46 *	862.34 ± 56.08 *
**IR+40** μM **Cur**	**74.25 ± 16.94** ^**#**^	**1291.05 ± 113.05** ^**#**^	**1369.34 ± 105.34** ^**#**^	**969.78 ± 87.49** ^**#**^
**IR+40μM Cur Hydrogel**	**81.93 ± 8.33** ^**#**^	**1481.23 ± 122.45** ^**#**^	**1527.57 ± 144.28** ^**#**^	**1149.78 ± 94.26** ^**#**^
**IR+40 Hydrogel**	**65.68 ± 18.91** ^***NS***^	**1108.32 ± 101.35** ^***NS***^	**1271.34 ± 101.76** ^***NS***^	**871.89 ± 76.32** ^***NS***^
**IR+40μMCur Hydrogel+AG490**	**63. 74 ± 22.45** ^***NS***^	**1089.34 ± 110.15** ^***NS***^	**1289.67 ± 121.54** ^***NS***^	**898.23 ± 85.12** ^***NS***^

*p < 0.05 vs sham; #*p* < 0.05 vs IR; *ns* nonsignificant

RETRACTED

**Table 2:** Detection of biochemical indexes in myocardial tissues

Group	SOD	CAT	GPX	GR
**Sham**	**153.86 ± 13.67**	**47.45 ± 3.79**	**67.39 ± 4.55**	**51.42 ± 4.93**
**IR**	48.38 ± 25.49 *	13.45 ± 1.72 *	23.29 ± 4.43 *	15.83 ± 1.33 *
**IR+40 μM Cur**	**94.25 ± 8.88** ^**#**^	**22.15 ± 2.62** ^**#**^	**44.37 ± 3.86** ^**#**^	**39.58 ± 13.55** ^**#**^
**IR+40μMCur Hydrogel**	**135.43 ± 11.35** ^**#**^	**38.93 ± 3.06** ^**#**^	**52.98 ± 4.93** ^**#**^	**44.78 ± 11.25** ^**#**^
**IR+40 Hydrogel**	**50.21 ± 32.16** ^***NS***^	**14.76 ± 1.87** ^***NS***^	**24.18 ± 2.76** ^***NS***^	**16.90 ± 2.92** ^***NS***^
**IR+40μMCur Hydrogel+AG490**	**61.42 ± 21.89** ^***NS***^	**16.31 ± 2.90** ^***NS***^	**27.37 ± 4.98** ^***NS***^	**18.43 ± 4.69** ^***NS***^

*p < 0.05 vs sham; #*p* < 0.05 vs IR; *ns* nonsignificant

**Table 3:** The activity of Ca^2+^ ATPase and Na^+^-k^+^-ATPase

Group	Ca^**2+**^ ATPase (μmol mg^**−1**^ h^**−1**^)	Na^**+**^-k^**+**^-ATPase (μmol mg^**−1**^ h^**−1**^)
**Sham**	**1.65 ± 0.14**	**3.28 ± 0.25**
**IR**	0.594 ± 0.05 *	1.274 ± 0.15 *
**IR+40μM Cur**	**0.874 ± 0.07** ^**#**^	**2.064 ± 0.19** ^**#**^
**IR+40μMCur Hydrogel**	**1.214 ± 0.11** ^**#**^	**2. 664 ± 0.25** ^**#**^
**IR+40 Hydrogel**	**0.601 ± 0.09** ^***NS***^	**1.358 ± 0.23** ^***NS***^
**IR+40μMCur Hydrogel+AG490**	**0.681 ± 0.11** ^***NS***^	**1.562 ± 0.14** ^***NS***^

*p < 0.05 vs sham; #*p* < 0.05 vs IR; *ns* nonsignificant

Left ventricular ejection fraction (EF) and left ventricular shortening fraction (FS) were detected by echocardiography. The results showed that cur-hydrogel could restore the cardiac function of model rats (Fig. 6a, b). The results of Evans blue staining showed that cur-hydrogel reduced the area of myocardial infarction (Fig. 6c). Treated with AG490, the EF and FS was decreased (Fig. 6a, b), and the area of myocardial infarction was increased (Fig. 6c).

**Fig. 6:** cur-hydrogel was better than curcumin in improving myocardial ischemia-reperfusion injury in rats**. a** Ejection fraction (EF%) and **b** fractional shortening (FS%) examined by echocardiography. *n* = 5, *p < 0.05; **p < 0.05; *ns* = nonsignificant. **c** Evans blue staining statistical chart of myocardial infarction area. *n* = 5, *p < 0.05; **p < 0.05; *ns* = nonsignificant. **d** HE and Masson staining of rat myocardial tissue (Bar = 40 μm). **e** TUNEL staining and statistical chart. (Bar = 40 μm) *n* = 5, *p < 0.05; **p < 0.05; *ns* = nonsignificant. **f** Protein level of JAK2/STAT3 by western blotting. *n* = 3, *p < 0.05; **p < 0.05; *ns* = nonsignificant

The myocardial tissue of rats was stained with HE and collagen was stained with Masson. The results showed that cur-hydrogel could restore the orderly arrangement of cardiomyocytes and inhibit the excessive deposition of collagen, AG490 blocked the therapeutic effect of curcumin hydrogel (Fig. 6d).

RETRACTED

Tissue TUNEL staining showed that, consistent with the results in vitro, heart injury led to the increase of apoptosis, curcumin could reduce the occurrence of apoptosis to some extent, but cur-hydrogel had better effect. However, AG490 promoted apoptosis of rat heart cells (Fig. 6e).

JAK2/STAT3 is an important intracellular signal transduction pathway, which involves a variety of pathological and physiological processes such as apoptosis, cell proliferation and differentiation. Western blot detection of myocardial homogenate showed that cur-hydrogel activated JAK2/STAT3 signal pathway in rat cardiomyocytes and played a role in myocardial protection. After blocking the JAK2/STAT3 pathway with AG490, the therapeutic effect of curcumin hydrogel disappeared (Fig. 6f). The above results showed that the effect of cur-hydrogel was better than that of curcumin.

## Discussion

Cardiac rational ventricular remodeling caused by myocardial infarction is one of the most common clinical causes of heart failure, which accelerates researchers’ efforts to develop new treatments and techniques to inhibit ventricular remodeling after myocardial infarction [17]. Among all kinds of biomaterials, injectable hydrogel has the advantages of good biocompatibility, degradability, high water solubility, and injectability, so it has a good development prospect and research value in the repair and treatment of myocardial infarction. Simple injection of hydrogel can provide mechanical support and structural filling for the damaged cardiac structure; increase the thickness of the ventricular wall in the infarcted area to prevent the ventricular wall from gradually thinning, dilating, or even rupturing; and improve cardiac function [18]. It can also be used as a carrier for carrying cytokines such as TIMP-3, VEGF, or FGF-2 and drug delivery [19, 20].

RETRACTED

Curcumin is an effective ingredient of turmeric, a traditional Chinese medicine, and has been used in China for thousands of years. Current studies have shown that it has a good protective effect on cardiovascular diseases, including diabetic cardiomyopathy [21], hypertension [22], cardiac hypertrophy [23], myocardial ischemia/reperfusion [24], and heart failure [25]. In addition, curcumin inhibits the progression of cardiomyocyte hypertrophy, apoptosis, and fibrosis by reducing inflammation and oxidative damage in cardiomyocytes and general heart tissue [26]. Curcumin is a known P300 inhibitor, in the rat model of diabetic cardiomyopathy, and curcumin can improve cardiac contractile function by inhibiting cardiomyocyte hypertrophy and cardiac fibrosis and reduce the expression of TGF-β1 [27]. Oral curcumin can reduce the progression of myocardial fibrosis induced by angiotensin II in rats, and this protective effect is related to the decrease of TGF-β1 expression and smad2/3 phosphorylation level in rat heart [28]. This study further confirmed that curcumin released from hydrogel can reduce the formation of reactive oxygen species, restore mitochondrial function, improve cardiac function, inhibit myocardial apoptosis, and activate JAK2/STAT3 pathway.

Previous studies have shown that curcumin is linked to the peptide to form compound I, which can greatly improve its water solubility, and the solubility in PBS can reach 10 mg/ml, showing a more effective anti-tumor effect [29]. In this study, we successfully prepared curcumin small molecular peptide hydrogel. Hydrogel can improve the water solubility and bioavailability of curcumin. Small peptide hydrogel can be degraded naturally in vivo, and the degradation product is small molecular amino acid, which is needed by the body and has high histocompatibility and safety. It can be used as a good extracellular matrix repair material to provide mechanical and functional support for left ventricular wall and improve cardiac structure and function.

JAK2/STAT3 is an important intracellular signal transduction pathway, which plays an important role in cellular stress, regulation of immunity, proliferation, apoptosis, inflammation, and tumor [30]. In myocardial tissue, JAK2/STAT3 signal pathway is closely related to the protective effect of myocardium. Studies have shown that JAK2/STAT3 activation inhibited cardiomyocyte apoptosis [31].

## Conclusions

In general, our study showed that cur-hydrogel could reduce cardiomyocyte apoptosis, ROS formation and mitochondrial damage in vitro, and the effect was better than that of curcumin. Compared with curcumin, cur-hydrogel can effectively improve cardiac function (FS,EF), inhibit left ventricular dilatation, inhibit ventricular remodeling and collagen synthesis, and activate JAK2/STAT3 pathway to protect injured myocardium in rat ischemia-reperfusion model, which may become a feasible scheme for clinical treatment of myocardial infarction.

RETRACTED

## Data Availability

The datasets used and analyzed during the current study are available from the corresponding author on reasonable request.

## Abbreviations

IRI: Ischemia-reperfusion injury
cur-hydrogel: Curcumin-hydrogel
LC-MS: Liquid chromatography-mass spectrometry
SOD: Superoxide dismutase
CAT: Catalase
GPX: Glutathione peroxidase
GR: Glutathione reductase

## References

[1] Ibanez B, Heusch G, Ovize M, Van de Werf F (2015). Evolving therapies for myocardial ischemia/reperfusion injury. J Am Coll Cardiol.

[2] Vogel B, Mehta SR, Mehran R (2017). Reperfusion strategies in acute myocardial infarction and multivessel disease. Nat Rev Cardiol.

[3] Liu Y, Xu J, Wu M, Kang L, Xu B (2020). The effector cells and cellular mediators of immune system involved in cardiac inflammation and fibrosis after myocardial infarction. J Cell Physiol.

[4] Yang Y, Zhou Q, Gao A, Chen L, Li L (2020). Endoplasmic reticulum stress and focused drug discovery in cardiovascular disease. Clin Chim Acta.

[5] Duan W, Yang Y, Yan J, Yu S, Liu J, Zhou J (2012). The effects of curcumin post-treatment against myocardial ischemia and reperfusion by activation of the JAK2/STAT3 signaling pathway. Basic Res Cardiol.

[6] Pang XF, Zhang LH, Bai F, Wang NP, Ijaz Shah A, Garner R (2015). Dual ACE-inhibition and angiotensin II AT1 receptor antagonism with curcumin attenuate maladaptive cardiac repair and improve ventricular systolic function after myocardial infarctionin rat heart. Eur J Pharmacol.

[7] Yao QH, Wang DQ, Cui CC, Yuan ZY, Chen SB, Yao XW (2004). Curcumin ameliorates left ventricular function in rabbits with pressure overload: inhibition of the remodeling of the left ventricular collagen network associated with suppression of myocardial tumor necrosis factor-alpha and matrix metalloproteinase-2 expression. Biol Pharm Bull.

[8] Yu W, Wu J, Cai F, Xiang J, Zha W, Fan D (2012). Curcumin alleviates diabetic cardiomyopathy in experimental diabetic rats. PLoS One.

[9] Sunagawa Y, Sono S, Katanasaka Y, Funamoto M, Hirano S, Miyazaki Y (2014). Optimal dose-setting study of curcumin for improvement of left ventricular systolic function after myocardial infarction in rats. J Pharmacol Sci.

[10] Saeidinia A, Keihanian F, Butler AE, Bagheri RK, Atkin SL, Sahebkar A (2018). Curcumin in heart failure: a choice for complementary therapy?. Pharmacol Res.

RETRACTED

[11] Gorabi AM, Hajighasemi S, Kiaie N, Rosano GMC, Sathyapalan T, Al-Rasadi K (2020). Anti-fibrotic effects of curcumin and some of its analogues in the heart. Heart Fail Rev.

[12] Wahlstrom B, Blennow G (1978). A study on the fate of curcumin in the rat. Acta Pharmacol Toxicol (Copenh).

[13] Peng JR, Qian ZY (2014). Drug delivery systems for overcoming the bioavailability of curcumin: not only the nanoparticle matters. Nanomedicine (Lond).

[14] Hatcher H, Planalp R, Cho J, Torti FM, Torti SV (2008). Curcumin: from ancient medicine to current clinical trials. Cell Mol Life Sci.

[15] Luo Z, Zhang S (2012). Designer nanomaterials using chiral self-assembling peptide systems and their emerging benefit for society. Chem Soc Rev.

[16] Liu J, Liu J, Xu H, Zhang Y, Chu L, Liu Q (2014). Novel tumor-targeting, self-assembling peptide nanofiber as a carrier for effective curcumin delivery. Int J Nanomedicine.

[17] Gallagher G, Menzie S, Huang Y, Jackson C, Hunyor SN (2007). Regional cardiac dysfunction is associated with specific alterations in inflammatory cytokines and matrix metalloproteinases after acute myocardial infarction in sheep. Basic Res Cardiol.

[18] Radhakrishnan J, Krishnan UM, Sethuraman S (2014). Hydrogel based injectable scaffolds for cardiac tissue regeneration. Biotechnol Adv.

[19] Skardal A, Murphy SV, Crowell K, Mack D, Atala A, Soker S (2017). A tunable hydrogel system for long-term release of cell-secreted cytokines and bioprinted in situ wound cell delivery. J Biomed Mater Res B Appl Biomater.

[20] Norouzi M, Nazari B, Miller DW (2016). Injectable hydrogel-based drug delivery systems for local cancer therapy. Drug Discov Today.

[21] Li K, Zhai M, Jiang L, Song F, Zhang B, Li J (2019). Tetrahydrocurcumin ameliorates diabetic cardiomyopathy by attenuating high glucose-induced oxidative stress and fibrosis via activating the SIRT1 pathway. Oxidative Med Cell Longev.

[22] Vamanu E, Gatea F, Sarbu I, Pelinescu D. An in vitro study of the influence of *Curcuma longa* extracts on the microbiota modulation process, in patients with hypertension. Pharmaceutics. 2019;11(4):191.10.3390/pharmaceutics11040191PMC652307431003502

[23] Liu R, Zhang HB, Yang J, Wang JR, Liu JX, Li CL (2018). Curcumin alleviates isoproterenol-induced cardiac hypertrophy and fibrosis through inhibition of autophagy and activation of mTOR. Eur Rev Med Pharmacol Sci.

[24] Mokhtari-Zaer A, Marefati N, Atkin SL, Butler AE, Sahebkar A (2018). The protective role of curcumin in myocardial ischemia-reperfusion injury. J Cell Physiol.

[25] Shimizu K, Sunagawa Y, Funamoto M, Wakabayashi H, Genpei M, Miyazaki Y (2020). The synthetic curcumin analogue GO-Y030 effectively suppresses the development of pressure overload-induced heart failure in mice. Sci Rep.

RETRACTED

[26] Zeng C, Zhong P, Zhao Y, Kanchana K, Zhang Y, Khan ZA (2015). Curcumin protects hearts from FFA-induced injury by activating Nrf2 and inactivating NF-kappaB both in vitro and in vivo. J Mol Cell Cardiol.

[27] Bugyei-Twum A, Advani A, Advani SL, Zhang Y, Thai K, Kelly DJ (2014). High glucose induces Smad activation via the transcriptional coregulator p300 and contributes to cardiac fibrosis and hypertrophy. Cardiovasc Diabetol.

[28] Pang XF, Zhang LH, Bai F, Wang NP, Garner RE, McKallip RJ (2015). Attenuation of myocardial fibrosis with curcumin is mediated by modulating expression of angiotensin II AT1/AT2 receptors and ACE2 in rats. Drug Des Devel Ther.

[29] Yang C, Wang Z, Ou C, Chen M, Wang L, Yang Z (2014). A supramolecular hydrogelator of curcumin. Chem Commun (Camb).

[30] Villarino AV, Kanno Y, O'Shea JJ (2017). Mechanisms and consequences of Jak-STAT signaling in the immune system. Nat Immunol.

[31] Oshima Y, Fujio Y, Nakanishi T, Itoh N, Yamamoto Y, Negoro S (2005). STAT3 mediates cardioprotection against ischemia/reperfusion injury through metallothionein induction in the heart. Cardiovasc Res.

